The article "Lateral Ventricular Volume Asymmetry and Optic Nerve Sheath Diameter Predict Intracranial Pressure in Traumatic Brain Injury Patients" was retracted in 2023. Reasons: signs of a paper mill; suspected computer-generated content; unreliable results or conclusions; concerns about the data.

# Lateral Ventricular Volume Asymmetry and Optic Nerve Sheath Diameter Predict Intracranial Pressure in Traumatic Brain Injury Patients

**DOI:** 10.1155/2022/9808334

**Published:** 2022-05-13

**Authors:** Yang Wang, Ziming Yuan, Zuoyan Zhang, Jiawei Shang, Mingna Li, Wei Wang

**Affiliations:** Department of Critical Care Medicine, Shanghai Jiao Tong University Affiliated Sixth People's Hospital, Shanghai 200030, China

## Abstract

**Background:**

Various noninvasive methods of intracranial pressure (ICP) measurement have been proposed. Each has unique advantages and limitations. This study was aimed at investigating the relationships between lateral ventricular asymmetry on admission computed tomography, optic nerve sheath diameter (ONSD), and ICP in traumatic brain injury (TBI) patients.

**Methods:**

A prospective observational study was conducted in the patients admitted to our department between October 2018 and October 2020. 20 patients with moderate-severe TBI with a Glasgow Coma Scale of 3–12 were enrolled. Lateral ventricle volume (LVV) value measurements were conducted using ITK-SNAP software. The lateral ventricular volume ratio (LVR) was quantified by dividing the larger LVV by the smaller.

**Results:**

ONSD and LVR had a good correlation with ICP. Admission LVR of >1.735 was shown to have a sensitivity of 90.9% and a specificity of 88.9% for prediction of ICP increase (AUC = 0.879; standard error = 0.091; 95% CI = 0.701 to 1.0; significance level *p* < 0.004). Admission ONSD of >5.55 mm was shown to have a sensitivity of 81.8% and a specificity of 88.9% for prediction of ICP increase (AUC = 0.919; standard error = 0.062; 95% CI = 0.798 to 1.0; significance level *p* < 0.002). Combining the ONSD and LVR, the sensitivity could be improved to 90.9% in parallel test, and the specificity could be improved to 100% in serial test.

**Conclusion:**

ONSD and LVR measurements can diagnose elevated ICP in traumatic brain injury patients. ONSD combining with LVR may further improve the diagnostic evaluation.

## 1. Introduction

Severe trauma is a notable major global public health problem, causing about approximately 1 in 10 mortalities and contributing to more than 5.8 million deaths annually worldwide [1]. Early evaluation of prognostic factors is crucial for decision-making, which is related to further treatment. One of the common and dangerous complications of brain injury is intracranial hypertension, which contributes to secondary brain injury. Severity and duration of intracranial hypertension are related to patient outcome [2]. Elevated intracranial pressure (sustained pressure greater than 20 mm Hg) is always associated with adverse clinical outcomes in traumatic brain injury (TBI) patients with neurologic impairment. At present, invasive intracranial pressure (ICP) monitoring is considered the gold standard because of its accuracy and high sensitivity; however, it requires strict neurosurgical settings and is associated with potential complications such as infection, bleeding, and brain lesions. Hence, the demand for a safe, accurate, and noninvasive ICP measurement method is extremely high. Although various methods have been put forward, each method has its own advantages and limitations. Most authors demonstrated good correlation with invasive ICP for many of these methods, in particular, eyeball ophthalmic artery method, MR method by Alperin, arterial TCD, and the TMD method [3]. However, most of these techniques are not easily available in clinical practice. All the noninvasive methods have the common disadvantage, that is, not accurate enough to replace the traditional invasive techniques. Most of the noninvasive techniques are affected by different operator-dependent factors, and in some cases, they cannot be applied to clinical practice [4–6]. Currently, bedside optic nerve sheath diameter (ONSD) assessment has been widely used to screen for increased ICP [7, 8]. Multiple studies have demonstrated a direct correlation between widened ONSD and elevated ICP in patients with severe head injury and intracranial bleeding. However, despite reliable high sensitivity and specificity, it is evasive to determine the consistent ONSD cutoff value for predicting ICP greater than 20 mmHg. At present, the optimal cutoff value given by many studies is ranging from 5 to 6.2 mm [9–11]. Despite recent improvements of imaging methods and neurobiomarkers, computed tomography (CT) is still the first-line tool for diagnosis, clinical treatment, and prognosis evaluation of patients with intracranial hemorrhage. A recent study indicated that the development of midline shift (MLS) in patients with traumatic brain injury can be predicted by lateral ventricular volume (LVV) asymmetry, induced by ipsilateral ventricular compression [12]. Nonetheless, noninvasive ICP measurement remains inadequate to replace invasive ICP monitoring [3]. We found that most studies used ONSD or LVV asymmetry alone, rather than a combination of the two. In this study, we aimed to inspect the role of ONSD and LVV asymmetry in diagnosing elevated ICP. In addition, we investigated the relationship between ONSD and LVV asymmetry.

## 2. Materials and Methods

### 2.1. Participants

We conducted a prospective observational study of patients admitted to our department between October 2018 and October 2020. We enrolled blunt moderate-severe TBI patients (with a Glasgow Coma Scale of 3–12) admitted to our ICU. A head CT was performed on admission to confirm the diagnosis. The exclusion criteria were as follows: (1) lesions that may cause intracranial hemorrhage such as intracranial tumors and aneurysms; (2) bilateral intracranial hemorrhage; (3) lack of data, such as baseline GCS score; (4) previous ocular and/or optic nerve diseases; (5) lack of ICP monitoring; and (6) age less than 18 years.

### 2.2. Treatments

Patients were clinically managed in accordance with international guidelines. The decision whether to place the invasive ICP monitor was made by the treating neurosurgeon based on Brain Trauma Foundation guidelines [13]. These guidelines are mainly based on the clinical status of patients on arrival (i.e., clinical deterioration with consciousness level decreased or rapid neurological function deteriorated) and neuroradiological findings (i.e., midline shift and impelling herniation).

### 2.3. Study Data

Study data included ICP value and head CT images and ONSD values. ONSD was measured in the neurological intensive care unit within 24 h after surgery. ICP values were recorded by an ICU doctor. ONSD and LVV values were obtained by ultrasound and CT, respectively, and the operators were blinded to the patient's ICP values.

ONSD measurements were done using the Philips Sparq ultrasound with the patient in a supine position. Patients were undergoing procedural sedation and analgesia with a continuous infusion of propofol or midazolam and fentanyl. Place conductive gel on tightly closed eyelids. Gently place the 12-4 MHz linear probe horizontally on the upper eyelid to form an axial cross-sectional image of the optic nerve, which can be seen longitudinally at the widest diameter of the orbit. The optic nerve sheath diameter was measured 3 mm behind the retina. Then, repeat the measurement on the other eye [14], each eye was measured 3 times, and the average value of 6 measurements was recorded. Not until the image processing and measuring, the provider was blinded to ICP measurements. ONSD values were measured by a physician who received one month of training in optic nerve sheath ultrasonography. For noninvasive ICP evaluation, ICP value remains to keep in a nonfluctuating state (<10% variation) for at least 30 min without requiring specific ICP-driven treatment, sputum aspiration, or other physical interventions. Head CT (Brilliance ICT, Philips Healthcare) was performed in all study patients on admission. CT acquisition parameters: 5 mm slice thickness, 120 kVp, 300 mAs, and 512∗512 pixels field of view.

ITK-SNAP software [open source] (version 3.6.0-RC1; http://www.itksnap.org) was used to measure LVV. LVV was realized by digital imaging and communications in patient's medicine images. According to the CT slices that contained the ventricles, we used the “freehand drawing style—polygon” of the “polygon inspector” modules to manually paint out the left and right lateral ventricles. For lateral ventricle three-dimensional reconstruction and volume estimation, choroid plexus and intraventricular hemorrhage were included in the outlines [12]. After segmenting and modeling the ventricle, the information about volume and mean CT value was calculated automatically (Figure 1). In order to quantitatively determine the asymmetry of LVV, the larger LVV is divided by the smaller LVV to quantify the lateral ventricular volume ratio (LVR), which terms the LVV ratio (LVR). The LVR was calculated for each TBI patient.

### 2.4. Consent

This study was approved by our ethics committee. Informed written consent was obtained from all patients or their families.

### 2.5. Statistical Analysis

SPSS software (version 22) was used for statistical analysis. A single sample K-S test was used to test the data normality. The continuous variables conforming to normal distribution were expressed as mean ± standard deviation (x ± s), while the data not in accordance with the normal distribution were expressed as median (*m*) and interquartile interval (IQR). Receiver operating characteristic (ROC) curve was performed to determine the optimal ONSD and LVR cutoff point to detect high ICP. All statistical tests were two-tailed. The significant level is set at 0.05.

## 3. Results

A total of 34 patients were screened and 20 enrolled (Table 1).

The average LVR for all evaluated TBI patients (*n* = 20) on admission scans was 2.6445 (SD = 2.27286); the median ICP was 22.75 mmHg (range 14-36). The value of baseline LVR in predicting elevated intracranial pressure was confirmed by ROC analysis (AUC = 0.879; standard error = 0.091; 95% CI = 0.701 to 1.0; significance level *p* (area = 0.5) <0.004). The optimized baseline LVR cutoff point was 1.735, and it had a sensitivity of 90.9% and specificity of 88.9% (Figure 2).

The mean diameter for the total of 20 US-ONSD readings was, respectively, 5.50 ± 0.65 mm and 5.54 ± 0.82 mm, for the left and right eyes. Correlation analysis showed that the mean ONSD was positively correlated with intracranial pressure, and the difference was statistically significant (*p* < 0.05). The optimized baseline ONSD cutoff point was 5.55 mm. Admission ONSD of >5.55 mm was shown to have a sensitivity of 81.8% and a specificity of 88.9% for prediction of intracranial pressure increase (AUC = 0.919; standard error = 0.062; 95% CI = 0.798 to 1.0; significance level *p* (area = 0.5) <0.002) (Figure 2).

When ONSD and LVR were used in combination, the results yielded a high sensitivity of 90.9% and specificity of 100%, with the AUC 0.97 (95% CI 0.901-1.0). Further tests revealed that combining ONSD and LVR in parallel test, the sensitivity could be improved to 81.8% and the specificity was 100%. On the meanwhile, the specificity was improved to 100%, with a sensitivity of 90.9% in serial test (Table 2).

## 4. Discussion

This study examined the association of LVV asymmetry on head CT at admission and ONSD measured on ultrasound with elevated ICP in 20 traumatic brain injury patients. Our findings suggest that ONSD measured on ultrasound is an excellent noninvasive diagnostic biomarker for ICP. Robba et al. showed [4] that ONSD was the best ultrasound-based method of estimating ICP. Similarly, a recent meta-analysis [9] that included 7 prospective studies showed that ultrasonographic ONSD may be helpful to assess intracranial hypertension when invasive equipment is not indicated or available, the area under the stratified summary ROC curve of 0.938. Our results (ROC curve of 0.919) support these findings. Chen et al. [15] proposed that measurement of ONSD may be potentially a noninvasive practice for dynamic, real-time monitoring of ICP fluctuation, extremely in the early phases. In their research, 95% of patients with a reduction in cerebrospinal fluid pressure showed an immediate decrease in ONSD, confirming that ONSD reacts to ICP in real time. The ONSD value is usually measured by an average of two eyes; asymmetric ONSD is possible, which may lead to using binocular averages to assess ICP may not be accurate. In addition, there is little data on ONSD asymmetry or the use of the maximum ONSD value between the eyes to assess elevated ICP. Naldi et al. [16] proposed that interocular ONSD asymmetry exists both in normal subjects and patients with elevated ICP. If asymmetry is present, it should be considered when estimating ICP. Therefore, we evaluated the relationship between the ratio of left and right eyes of ONSD and ICP and found that they were not correlated. Normal control group can be added to further research to prevent bias. Geeraerts et al. [14] published the ONSD cutoff value (5.86 mm) of pathological ICP; meanwhile, literature data showed that 90% of ONSD measurements were equal to or higher than this value, so do our articles.

At present, we know little about intracranial compensatory reserve. Depending on the study, 6.5-26% of patients who initially receive conservative treatment may eventually require surgery [17, 18]. For patients with chronic subdural hematoma [19], ICP may be within or close to the normal range, even in those with thick hematomas and/or midline shift. The prognostic value of intracranial hemorrhage was often studied using mass effect signs, perihematomal edema expansion, and MLS. In our study, LVR measurement was used as a simple approach to quantify lateral ventricle asymmetry. LVR may provide more detailed information concerning mass effect than hematoma volume alone. Several large clinical trials [20, 21] have focused on reducing hematoma dilatation through a rigorous treatment window; most of them occurs within 24 hours of the onset of ICH. LVV asymmetry is an indicator of brain deformities which may help detect underlying pathological features of asymmetry prior to midline displacement, and management objectives are not limited to the treatment window. Therefore, early detection and treatment of LVV asymmetry may be helpful to improve the prognosis. Tóth et al. [12], as we know, the first one to quantify the threshold of lateral ventricle asymmetry, reported that severe TBI patients with an LVR greater than 1.67 may subsequently develop MLS, which is consistent with the previous communications [22, 23]. Since patients with a high LVR and ONSD tended to have large hematoma volume and severe perihematomal edema, MLS was more likely to occur due to the increase of ICP. Therefore, these patients are more likely to benefit from early aggressive treatment such as surgical evacuation of the hematoma or administrated of megadose dehydrating agent. After all, the ultimate goal of treatment was to reduce ICP, which may avoid the appearance of subsequent ICP asymmetry. It is possible that ventricular asymmetry may be an early indicator of brain pathology. Increased intrahemispheric pressure due to hemorrhage or edema can cause compression of the ipsilateral ventricle, leading to a subfalcine hernia or falcine deformity. Alternatively, unilateral ventricular entrapment can cause ventricular enlargement and increased intrahemispheric pressure. This early evaluation index of asymmetric brain distortion may be clinically relevant and helpful to detect intracranial pathological changes before midline displacement occurs. As an early sign of elevated ICP, elevated LVR might be an independent predictor of poor prognosis in patients with intracranial hemorrhage [24].

Notably, we find that “ONSD+LVR” achieved high specificity and sensitivity for detecting elevated ICP. Therefore, we suggest that “ONSD+LVR” can be used to estimate ICP noninvasively.

To our knowledge, this is the first time that ONSD and LVR were used together to predict nICP. However, there are several limitations. First, the sample size was small, and it was conducted in a single center. Therefore, our findings may not be generalizable. In addition, it was not possible to completely blind the sonographer to patient details. Third, our study did not involve the normal control group, and there was a convenience to judge whether the measured LVR or ONSD was a normal variation or a pathological variation. Moreover, the vast majority of measurements were carried out within relatively well-controlled ICP; therefore, our findings cannot be extrapolated to patients with highly variable ICP.

## 5. Conclusion

In conclusion, the combination of ONSD and LVR methods showed a statistically significant improvement of AUC values compared with the ONSD or LVR method alone. Noninvasive measurement of ONSD and LVR can predict elevated ICP in traumatic brain injury patients. Diagnostic sensitivity and specificity are improved when the two methods are combined. However, further studies are needed to confirm and validate our findings.

## Figures and Tables

**Figure 1:** Admission computed tomography and LVV images of representative patients (a 60-year-old man was hospitalized for falling down with admission GCS 11) with high lateral ventricular volume ratio. (a) Computed tomographic view of the head demonstrating hematoma and lateral ventricular volume (LVV) asymmetry. (b) Segmentation of lateral ventricles and hematoma into different colors by use of ITK-SNAP software. Blue, left lateral ventricle; green, right lateral ventricle; red, hematoma. (c and d) Relationships between lateral ventricles and hematoma shown in front and superior views.

**Figure 2:** Receiver operating characteristic curve in TBI patient with ONSD and LVR for n-ICP diagnosis.

**Table 1:** Baseline characteristics of the patient cohort.

Characteristic	*N* (%) or median (IQR)
Total number	20
Male sex	15 (75.0%)
Age (years)	60.5 (51-67)
Height (cm)	173.5 (166.7–175.7)
Weight (kg)	71.0 (65.7–75)
Comorbidities	
Hypertension	8 (40%)
Alcohol abuse	1 (5%)
Smokers	9 (45%)
GCS at admission	8 (7–9.7)

GCS: Glasgow Coma Scale.

**Table 2:** Diagnostic performance of ONSD, LVR, and combination diagnostic test.

	AUC	95% CI		*P*	Sensitivity (%)	Specificity (%)	PPV (%)	NPV (%)
		Lower	Upper					
LVR	0.879	0.701	1.000	0.004	90.9	88.9	90.9	88.9
ONSD	0.919	0.798	1.000	0.002	81.8	88.9	90.0	80.0
Parallel test	0.843	0.651	1.000	0.01	90.9	77.8	83.3	87.5
Serial test	0.909	0.766	1.000	0.002	81.8	100	100.0	81.8
Predicted probability	0.970	0.901	1.000	<0.001	90.9	100.0	100.0	90.0

PPV: positive predictive value; NPV: negative predictive value.

## Data Availability

The data used to support the findings of this study are available from the corresponding author upon request.
